# Diet improvement for western corn rootworm (Coleoptera: Chrysomelidae) larvae

**DOI:** 10.1371/journal.pone.0187997

**Published:** 2017-11-17

**Authors:** Man P. Huynh, Lisa N. Meihls, Bruce E. Hibbard, Stephen L. Lapointe, Randall P. Niedz, Dalton C. Ludwick, Thomas A. Coudron

**Affiliations:** 1 Division of Plant Sciences, University of Missouri, Columbia, Missouri, United States of America; 2 Department of Plant Protection, Can Tho University, Can Tho, Vietnam; 3 Plant Genetics Research Unit, USDA-Agricultural Research Service, Columbia, Missouri, United States of America; 4 Horticultural Research Laboratory, USDA-Agricultural Research Service, Fort Pierce, Florida, United States of America; 5 Biological Control of Insects Research Laboratory, USDA-Agricultural Research Service, Columbia, Missouri, United States of America; University of Tennessee, UNITED STATES

## Abstract

The western corn rootworm (WCR), *Diabrotica virgifera virgifera* LeConte, is the most serious insect pest of corn (*Zea mays* L.) in the United States and parts of Europe, and arguably one of the world’s most expensive pests to control. Several diet formulations are currently used by industry and public researchers to evaluate WCR larvae in diet-toxicity bioassays. However, a publicly available diet that produces normative insects that are physiologically similar to WCR larvae reared on corn roots will accelerate development of management technologies. We report a new diet formulation that supports improved weight gain, larval development and survival compared with the only public diet for WCR that is currently available in the refereed literature. The formulation was created by using response surface methods combined with n-dimensional mixture designs to identify and improve the formulation of key ingredients. Weight gain increased two-fold, and survival and molting rates increased from 93% and 90%, respectively when reared on the public diet, to approximately 99% for both survival and molting at 11 days when reared on our new formulation. This new formulation provides a standardized growth medium for WCR larvae that will facilitate comparison of research results from various working groups and compliance with regulatory requirements.

## Introduction

The western corn rootworm (WCR), *Diabrotica virgifera virgifera* LeConte, is the most serious insect pest of maize in the United States and parts of Europe. The larval stage feeds primarily on maize roots and is responsible for the majority of damage caused by WCR. Adult WCR feed on the green silks of maize plants and may cause yield reduction at high densities if present prior to anthesis [1]. Crop losses and abatement efforts to minimize damage by corn rootworm have been estimated to reach $2 billion annually [2]. Management of WCR has continuously presented a challenge to industry and corn growers because WCR has developed resistance to management tactics including chemical insecticides [3–5], crop rotation [6,7], and transgenic maize which expresses insecticidal proteins derived from *Bacillus thuringiensis* (Bt) [8]. Presently, some level of field-evolved resistance has developed to all single-gene Bt proteins currently available for WCR management [9–11].

Research efforts to avert resistance development require some level of ability to rear WCR. Although a standardized rearing method for research and regulatory purposes is highly preferred [12], a standardized method has not been adopted for WCR and consequently both plant and diet rearing systems are currently used for bioassays. Life history parameters and toxicity results differ greatly across these systems, making comparisons difficult and limiting the extent to which results can be interpreted [13]. An artificial diet that supports normative development of WCR larvae (i.e., similar to that of WCR reared on maize root) would be a major advancement in achieving a standardized bioassay method.

The first artificial diet for *Diabrotica* species was formulated for the southern corn rootworm (SCR), *Diabrotica undecimpunctata howardi* Barber. The ease of rearing SCR made it an attractive substitute for WCR in experiments [14]. This agar-based diet with wheat germ and casein as the major nutritional components supported development from egg to adult but resulted in slower development and reduced fecundity compared to those reared on corn roots. Subsequent changes to the formulation [15,16] increased raw linseed oil and sucrose, and decreased antimicrobial agents and potassium hydroxide. These changes resulted in a diet that supported developmental rates for SCR that were similar to larvae reared on corn roots, but only after 6 generations of rearing on the diet, which suggests some formulation improvements were still possible.

Pleau et al. [17] formulated the only published diet for rearing WCR larvae, which was a modification of diets developed for SCR [14,16]. Several important differences were noted when adjusting the diet for WCR. Optimizing the pH, removing formalin and adding corn root powder nearly doubled the weight of WCR larvae compared with the SCR formulation [17]. This diet has been used in a diet-toxicity bioassay to evaluate baseline susceptibility of various WCR populations to a Cry3Bb1 toxin [18]. However, for a WCR diet to achieve its full potential of fulfilling the needs of researchers, regulatory agencies and industry, improvements will have to support diet bioassays sensitive enough to detect differences between susceptible and resistant insects, to support molting, to be publicly available, and ultimately, to obtain development similar to when WCR is reared on corn roots [13,19,20].

Formulation efforts for improving the artificial diet for SCR and WCR discussed above measured biochemical and/or physiological parameters to test the effect of changes in diet formulation on insect performance. Typically, diet components were changed one at a time and insect performance was assessed after each change following a lengthy feeding period. This traditional method to determine the effect of varying the doses of several components requires large factorial experiments resulting in a huge numbers of treatment combinations and parallel variation of variables, making it difficult to interpret the results [21]. However, the process of changing one-ingredient-at-a-time (OIAT) within a mixture is not capable of identifying an optimal blend of the ingredients because the effects of proportion and amount are confounded in factorial designs [22]. When the proportion of any ingredient is varied, the proportions of all remaining ingredients are also changed. For this reason, mathematical models were developed by Henri Scheffé [23] to deal specifically with the problem of modeling responses to mixtures, now commonly referred to as Scheffé models or Scheffé polynomials. Response surface modeling (RSM) and advanced software [24,25] have simplified the corresponding computations. The application of RSM based on multivariate geometric design for mixtures [25–28] is of great value for insect diet improvement and optimization.

Other insect diet formulations have been improved using multi-dimensional mixture designs [25] to help identify ingredients (i.e,. key ingredients) that have the greatest effect on insect development. A mixture experiment used to formulate a diet is a special type of response surface experiment [25,29] in which ingredients are mixture components as input variables, and life history traits as response measures. Mathematical equations can be derived that predict the impact of diet components on insect responses and in that manner used to generate formulation improvements. Validation experiments are conducted to verify that the new formulations result in the predicted performance improvements.

The objective of this research was to optimize the composition of ingredients in the Pleau et al. diet [17]. The approach used multivariate geometric mixture designs combined with response surface modeling [25] to identify and evaluate the proportion of the key components in the diet for improved larval performance (larval survival, development, and weight) while limiting diet contamination.

## Materials and methods

### Insects

WCR eggs (non-diapausing strain) were obtained from the USDA-ARS Plant Genetics Research Unit at Columbia, Missouri, in a Petri dish with 70 mesh sieved soil and incubated at a constant 25°C in darkness. After several larvae were observed to hatch, the remaining eggs were washed out of the soil using a technique described by Pleau et al. [17]. The soil was washed through a 60 mesh sieve with water. The remaining eggs were surface-treated first with undiluted lysol^®^ (Reckitt Benckiser, LLC, Parsippany, NJ) for 3 min and then triple rinsed with distilled water. Next, the eggs were treated with 10% formalin (product # HT501128, Sigma Aldrich, St. Louis, MO) for 3 min and then triple rinsed with distilled water. The eggs were pipetted onto a coffee filter paper (Pure Brew, Rockline Industries, Sheboygan, WI) held inside a 16 oz. Solo^®^ deli cup with a plastic lid (product #LG8RB-0090 and #DM16R-0090, Solo Cup Company, Lake Forest, IL) containing 5 to 6 vent holes made by a number zero insect pin, and incubated at 25°C until hatch.

### Diet preparation

The diet was prepared using a procedure modified from Pleau et al.[17]. All glassware and containers were sterilized with ca. 0.5% sodium hypochlorite or exposure to UV light for 5 minutes prior to use. Distilled water and agar (product #A7002, Sigma-Aldrich) were added to a 400 ml glass beaker. The solution was boiled in a microwave for 2 min and then poured into a blender (Hamilton Beach, Inc., Model 51101BZ). The agar solution was cooled to 65^o^ C and wheat germ (product #1661, Bio-Serv, Flemington, NJ), casein (product #1100, Bio-Serv), cellulose (product #3425, Bio-Serv), sucrose (product #04821721, MP Biomedicals, Santa Ana, CA), corn root powder (Monsanto, St Louis, MO), salt mix (product #F8680, Bio-Serv), vitamin mix (product #V1007, Sigma-Aldrich), methyl paraben (product #H5501, Sigma-Aldrich), cholesterol (product #C8503, Sigma-Aldrich), and sorbic acid (product #S1626, Sigma-Aldrich) were added to the blender and mixed thoroughly. The diet was poured into a 750 ml glass beaker containing a stir-bar and placed on a stirring hot plate (Thermo scientific, Cimarec^TM^). The mixture was held at 65°C and slowly stirred while adding other ingredients, i.e., linseed oil (product #430021, Sigma-Aldrich), wheat germ oil (product #W1000, Sigma-Aldrich), streptomycin (612240500, Across, Morris Plains, New Jersey), chlortetracycline (C4881, Sigma-Aldrich). Green food coloring (Bulter, Lancaster, PA) was added to improve visual contrast. The pH of the diet was adjusted to 9 by adding 10% KOH (w/v) (product #P250, Fisher Scientific, Fair Lawn, NJ) and monitored with indicator strips (Whatman). The molten diet was dispensed into wells (200 μl/well) of a 96-well immunoassay plate (product #3370, Corning Inc., Corning, NY) using a repeater pipette (Eppendorf repeater plus). The diet was placed in a biological safety cabinet (Nuaire, Biological safety cabinet) and allowed to cool and evaporate excess moisture for 30 min. All subsequent diet and insect transfers were done in the biological cabinet. Plates were stored in a refrigerator at 4°C and used within two weeks. Each formulation was pipetted into a randomly-assigned 12-well row on the plate. Eight different diet solutions were tested per plate. Each formulation was replicated at least 4 times. The response of 12 larvae was averaged and constituted a single replication in the analysis.

### Insect bioassays

Larvae were transferred onto the diet within in a sterile biological safety cabinet within 24 h of hatching. One larva was placed per well using a No. 1 paintbrush. The plate was covered with a sealing film (Excel scientific, Inc., Thermalseal RTS^RM^, TSS-RTQ-100) and a single vent hole was made over each well with an insect pin (size 0). The plates were held in the dark at 25°C. Larvae were checked daily. Surviving larvae from each formulation were collected and pooled within a replication after 7 or 11 days and stored in 95% ethanol. Collections made at 7 days were used to determine survival and weight differences and to allow comparison of our data with previously published data. Collections made at 11 days were used to determine differences in survival, weight and molting to the 2^nd^ instar. Diet contamination (fungal and bacterial), larval survival, and time of molt to second instar were recorded during the bioassay and dry larval weight was determined after the bioassay. For dry larval weight, excess ethanol was discarded, and the remaining ethanol was evaporated and the larvae dried in an oven (Blue M Therm Dry Bacteriological Incubator, Model #602752) at 50°C for two days. Dried larvae were weighed with a micro balance (Sartorius^TM^ Cubis^TM^, 6.6S).

### Experimental approach

An iterative approach was used to identify and optimize critical diet ingredients for specific response variables. An initial screening design [30] was used to identify ingredients with large effects on the measured responses from the 8 components of a previously published diet [17]. These ingredients were carried forward to the second phase.

The dimensionality of mixture designs can be expressed as *n*-1 dimensions where *n* is the number of components [22]. Therefore, the screening design of 8 ingredients is referred to as a 7-dimensional design space. Polynomial equations were generated to describe the impact of important ingredients on larval weight, proportion of larvae undergoing a successful molt, survival and diet contamination. The contribution of 2 lipid components (wheat germ oil and linseed oil) were tested in a separate experiment to confirm results produced in the 7-dimensional study. A reduced 3-dimensional design (4 ingredients) was used to identify an optimal formulation of the 4 ingredients identified in the screening design [25]. Optimization in this context refers to the best combination of the ingredients studied. The predicted optimal blend of 4 ingredients was then validated in a separate experiment in comparison with the Pleau et al. diet [17].

#### Screening design

The diet ingredients used in this study included 17 ingredients used in a previously published formulation for WCR larvae [17] plus wheat germ oil (Table 1). The screening design was formulated to simultaneously vary 8 diet components: wheat germ, casein, corn root powder, cellulose, sucrose, linseed oil, wheat germ oil and agar. Other ingredients (vitamin and salt mixtures, preservatives and antibiotics) were kept constant at the level reported by Pleau et al. [17]. No attempt was made to deconvolute two commonly used insect diet supplements, Wesson salt mix and Vanderzant vitamin mix [25]. A 7-dimensional mixture screening design was created with Design-Expert (v.10.0, Stat-Ease, Inc., Minneapolis, MN) resulting in 22 design points including vertex, center, 7-blend, and axial check blend points (Table 2) [24]. The resulting simplex, linear design had 7 model, 9 lack of fit and 5 pure error degrees of freedom [31]. Duplication of design points was sufficient to estimate pure error across the design space and to attain near uniform leverage for all design points [32].

**Table 1:** Component that were proportionally varied or held constant in diets used to rear western corn rootworm larvae.

Variable components	Constant components
1. Agar	1. Chlortetracycline (10 mg/ml)
2. Casein	2. Distilled water
3. Cellulose	3. Cholesterol
4. Corn root powder	4. Food coloring
5. Linseed oil	5. Methyl paraben
6. Sucrose	6. Potassium hydroxide (10%)
7. Wheat germ, ground	7. Sorbic acid
8. Wheat germ oil	8. Streptomycin (12.8 mg/ml)
	9. Vanderzant vitamin mix
	10. Wesson's salt mix

**Table 2:** Diet blends of 8 components varied in a 7-dimensional, mixture screening design to rear western corn rootworm larvae.

Diet blend #	Agar (g)	Sucrose (g)	Wheat germ (g)	Casein (g)	Cellulose (g)	Corn root (g)	Linseed oil (μl)	Wheat germ oil (μl)
1	1	1	7.02	5	1	1	0	0.05
2	1	1	3.97	5	5	0	0.05	0.05
3	2.89	2.89	3.97	2.89	2.89	0.50	0.02	0.025
4	1	5	4.02	1	5	0	0.05	0
5	5	1	8.02	1	1	0	0.05	0
6	1	1	10	1	3.02	0	0	0.05
7	5	5	1	3.02	1	1	0	0.05
8	1	1	7.07	5	1	1	0	0
9	1	1	8.02	5	1	0	0	0.05
10	5	5	1	1	4.02	0	0	0.05
11	2.89	2.89	3.97	2.89	2.89	0.50	0.025	0.025
12	2.89	2.89	3.97	2.89	2.89	0.50	0.025	0.025
13	5	4.02	1	5	1	0	0.05	0
14	1	1	10	1	2.02	1	0	0.05
15	3.01	1	10	1.06	1	0	0	0
16	2.89	2.89	3.97	2.89	2.89	0.50	0.025	0.025
17	1	5	1	3.07	5	1	0	0
18	2.89	2.89	3.97	2.89	2.89	0.50	0.025	0.025
19	5	1	3.02	1	5	1	0.05	0
20	5	1	1	2.97	5	1	0.05	0.05
21	1	5	6.97	1	1	1	0.05	0.05
22	1	5	6.97	1	1	1	0.05	0.05

#### 4-component mixture design

The 4 ingredients responsible for the greatest improvement in WCR larval weight in the screening design (not including lipid components) were used to construct an I-optimal mixture design sufficient to satisfy a Scheffé special cubic polynomial response surface model (Table 3) [30]. The design consisted of 21 design points with 13 model, 2 lack of fit and 5 pure error degrees of freedom. A set of equations was derived that described insect responses (i.e., survival, molt from 1^st^ to 2^nd^ instar, and weight) at set time points (i.e., 7 day or 11 day) to varying blends of 4 key ingredients (wheat germ, casein, corn root powder and cellulose). Optimal blends were predicted using a simplex hill-climbing algorithm included in Design-Expert™ software [25]. The equations enabled us to calculate the best optimal formulation based on desirable criteria (e.g. molt, weight, survival, contamination).

**Table 3:** Diet blends of 4 ingredients varied in a three-dimensional mixture design to rear western corn rootworm larvae.

Diet blend #	Sucrose (g)	Wheat germ (g)	Casein (g)	Corn root powder (g)
1	5	4	0	3
2	5	1.2	2.8	3
3	0	8.8	0.2	3
4	0	5.3	5	1.7
5	3.5	2.9	3.9	1.7
6	1.2	10	0	0.8
7	2.4	4.6	5	0
8	0	10	2	0
9	2.9	5	2.4	1.7
10	0	8.8	0.2	3
11	5	7	0	0
12	0	5.3	5	1.7
13	2.4	7.7	1.9	0
14	2.4	4.6	5	0
15	1	3.1	4.9	3
16	5	4	0	3
17	0	10	2	0
18	3	1	5	3
19	5	4.3	2.7	0
20	5	1	5	1
21	2.5	5.5	2.5	1.5

#### 2-component mixture design for lipid components

The 2 lipid ingredients, wheat germ oil and linseed oil, were used to construct an I-optimal mixture design consisting of 5 design points including center, vertex and axial check blend points (Table 4). Response surface models were generated to validate the results produced in the screening design and to illustrate the contribution of lipid components of the Pleau et al. diet.

**Table 4:** Diet blends of 2 lipid components varied in a 1-dimensional mixture design to rear western corn rootworm larvae.

Diet blend #	Wheat germ oil (μl)	Linseed oil (μl)
1	50	450
2	150	350
3	250	250
4	350	150
5	450	50

#### Diet optimization

A formulation for maximizing larval performance (survival, molting, and weight) was calculated with Design-Expert^TM^. This software used direct search methods [33] to maximize the desirability function [25,29].

#### Model evaluation

All three measures of larval performance (survival, molting, and weight) reared on the improved diet identified by the response surface mixture model were compared with those of larvae reared on the published WCR diet [17].

### Statistical analyses

Survival and molting data were generated by dividing the number of live larvae and successful larval molt from 1^st^ to 2^nd^ instar per replicate, respectively by the initial number of larvae infested and multiplying by 100 to obtain percentages. Weight data were generated by dividing total weight per replicate by the number of live larvae.

For each measured response of larval performance (larval survival, proportion of successful larval molts and larval weight), all possible models from the mean to quartic polynomial were calculated with Design Expert^®^. Initial model selection was based on criteria that included a lack of aliased terms, low residual values, low model *P*-value, nonsignificant lack of fit, low standard deviation, high R^2^, R^2^_adj_ and R^2^_pred_, close agreement between R^2^_adj_ and R^2^_pred_, and a low PRESS value. R^2^ is a measure of variation around the mean explained by the response surface model. R^2^ can become biased if extraneous model terms are introduced. Therefore, the adjusted-R^2^ (R^2^_adj_) decreases as the number of terms in the model increases if those additional terms do not increase the precision of the model [25]. PRESS is the prediction error sum of squares [34] calculated by removing a single observation from the response surface model, predicting that response point with the remaining *n*-1 observations, repeating this process for all observations, and then summing the squares of the *n* PRESS residuals [31]. If two or more models were satisfactory, then the most stringent one was chosen. The selected model was then further evaluated according to a battery of adequacy tests as described by Anderson and Whitcomb [24,35] and Lapointe et al. [25].

In the validation experiment, measured parameters of larval performance on the Pleau et al. diet and an improved diet at 7 and 11 days after infestation were analyzed as a randomized complete block design using PROC MIXED in SAS [36]. All percent variables were arcsine square-root transformed prior to the analysis to meet assumptions of normality and homoscedasticity.

## Results

### 8-component screening experiment

The screening design produced a significant linear response model for larval weight (*p* = 0.009, *F* = 4.44, d.f. = 7) by varying 8 diet components: agar, sucrose, wheat germ, casein, cellulose, corn root powder, wheat germ oil and linseed oil (Tables 1 and 2). We found a direct positive relationship between weight gain and proportion of casein, wheat germ, corn root and linseed oil, shown as a Piepel trace plot (Fig 1). Piepel trace plots estimate the effect of increasing the proportion of one component in relation to a reference blend while the relative proportions of all of the other diet components are kept constant [37]. In Fig 1, a linear model resulted in linear traces. The slope of the line indicates the direction and magnitude of the influence of the individual factors on the measured response variable, e.g., larval weight.

**Fig 1:** Piepel trace plot of larval weight deviation from a reference blend diet. Reference blend proportions: agar = 0.171, sucrose = 0.171, wheat germ = 0.267, casein = 0.171, cellulose = 0.171, corn root: 0.045, wheat germ oil = 0.002, linseed oil = 0.002. A: agar, B: sucrose, C: wheat germ, D: casein, E: cellulose, F: corn root, G: wheat germ oil, H: linseed oil.

The greatest increase in weight was seen with proportional increases of casein and wheat germ. In contrast, we found that weight decreased with increasing proportions of agar, cellulose, sucrose and wheat germ oil (Fig 1). The greatest decrease in weight was seen when the proportion of agar was increased. Given that six ingredients (i.e., wheat germ, casein, corn root, linseed oil, wheat germ oil and sucrose) had the greatest influence on larval weight, they were chosen for further experimentations. Wheat germ, casein, corn root and sucrose were used within a 4-component mixture design and wheat germ oil and linseed oil were used within a 2-component mixture design.

### 4-component mixture experiment

The 4-component mixture design yielded significant response surface models for all three measures of larval performance (survival, molt, and weight) by varying 4 diet components: wheat germ, casein, corn root powder and sucrose (Table 3), shown as Ternary plots (Fig 2). The ternary plots represent the universe of possible combinations of proportions of three components while proportions of other components (if applicable) are constant. In this case, prior knowledge constrained the amounts of certain diet ingredients resulting in the constrained regions shown in the response surfaces in Fig 2. The labelled isobars and color indicate the magnitude of the response variables in a dimension that can be envisioned as perpendicular to the page.

**Fig 2:** Predicted 3-D surface response plots for WCR larvae reared on different diets. (A) weight, (B) survival, and (C) molt, at 7 days post infestation. For (A) the proportion of corn root powder was constant at 0.27. For (B) and (C) the proportion of casein was constant at 0.27. Color bars display the magnitude of the measured response.

The mixture design produced a significant special cubic model for weight (*p*<0.001, *F* = 128.74, d.f. = 10). The model was improved by stepwise regression (reduced). R^2^, R^2^_adj_ and R^2^_pred_, (0.99, 0.99 and 0.95, respectively) were clustered with a difference <0.05. Lack-of-fit was not significant (Table 5). The response surface for weight gain indicated that casein was the most important component for maximizing larval weight. Wheat germ and corn root powder had a positive influence on weight while sucrose had a negative effect (Fig 2A). Interestingly, casein and corn root powder had an inverse blending effect (interaction), in which increasing proportion of casein with decreasing proportion of corn root powder resulted in an increase in weight (Fig 3A).

**Fig 3:** Nonlinear blending effects in the 4-component mixture experiment. (A) casein x corn root powder, (B) casein x sucrose, and (C) casein x wheat germ. Dotted lines indicate 95% confidence interval bands.

**Table 5:** *p*-values, regression coefficients and response surface model fitting diagnostic statistics for WCR larval responses to 4-component diet mixtures.

	Weight *p*-values	Regression coefficients	% Survival *p*-values	Regression coefficients	% Molt *p*-values	Regression coefficients
Model	<0.0001	-	0.0006	-	<0.0001	-
Linear mixture	<0.0001	-	0.0029	-	<0.0001	-
A	-	0.13	-	0.72	-	-2.17
B	-	0.05	-	0.97	-	-0.33
C	-	-0.13	-	0.02	-	-3.86
D	-	-0.67	-	0.65	-	1.28
A x B	0.1981	-1.88	-	-	0.0020	4.68
A x C	0.1999	0.16	-	-	<0.0001	12.61
A x D	0.0014	0.76	-	-	0.7000	-0.80
B x C	0.0029	0.48	-	-	<0.0001	8.12
B x D	0.0005	0.85	-	-	0.5689	-0.94
C x D	<0.0001	1.78	0.0020	4.19	0.0021	6.74
A x B x C	0.0105	1.42	-	-	0.0097	10.96
A x B x D	-	-	-	-	0.0052	9.47
Lack of fit	0.3901		0.6193		0.9866	
Model type	Special Cubic (reduced)		Quadratic (reduced)		Special Cubic (reduced)	
Transformation	N/A		N/A		Arcsin Sqrt (%molt+0.01)	
R^2^	0.9923		0.6869		0.9759	
R^2^_adj_	0.9846		0.6086		0.9465	
R^2^_pred_	0.9488		0.4464		0.8996	

A: sucrose, B: wheat germ, C: casein, D: corn root powder. Arcsin Sqrt: arcsine square root.

The best-fit model for survival was quadratic (*p* <0.001, *F* = 8.77, d.f. = 4). The model was improved by stepwise regression. R^2^, R^2^_adj_ and R^2^_pred_ (0.69, 0.61 and 0.45, respectively) were clustered and lack of fit was not significant (Table 5). Wheat germ and corn root powder were both influential in maximizing the number of larvae that survived at 7 days post infestation. In contrast, casein and sucrose at higher proportions had negative effects on larval survival rates (Fig 2B).

The mixture design produced a significant special cubic model for the percent of larvae that successfully completed a molt (*p*<0.001, *F* = 33.16. d.f. = 11). Percent molting was transformed by arcsine square root. The model was improved by stepwise regression. R^2^, R^2^_adj_ and R^2^_pred_ were 0.98, 0.95 and 0.90, respectively. Lack of fit was not significant (Table 5). Corn root powder had a very strong influence on the developmental rate (measured by time to molt). The percentage of larval molts increased with increasing proportion of corn root powder. Additionally, increased casein, wheat germ, and sucrose lowered molting rates (Fig 2C). Results also showed very strong antagonistic blending effects of casein x sucrose and casein x wheat germ, indicating that an increase in casein at higher proportions with decreasing proportions of sucrose or wheat germ resulted in decreased molting (Fig 3B and 3C).

There was an inverse relationship between weight, survival and molting when proportions of corn root powder, casein and wheat germ varied; shown as Piepel trace plots (Fig 4). The quadratic models describing the responses to the four-blend diet showed curvature and revealed nonlinear relationships between proportionality of some diet components and the response variable. Specifically, an increase in corn root powder up to a proportion of 2.7% (w/w) resulted in an increase in both molting and survival, but an increase in corn root powder higher than the proportion of 1.2% (w/w) resulted in a decrease in weight. However, a high proportion of casein had a positive effect on larval weight gain, but a negative effect both on molting and survival. An increase in casein up to the proportion of 3.8% (w/w) maximized larval weight whereas a decrease in casein below 1.8% (w/w) caused a decrease in molting. An increase in proportion of wheat germ up to the level of 6.3% (w/w) resulted in an increase in survival but higher proportions resulted in a decrease in weight and molting. In contrast, an increase in wheat germ above 3.5% (w/w) and 4.6% (w/w) resulted in a decrease in weight and molting, respectively. Consequently, the optimum proportion of corn root powder, casein and wheat germ for molting, survival and weight were different.

**Fig 4:** Piepel trace plots of weight, survival and molt deviation from a reference diet. (A) weight, (B) survival, and (C) molt. Reference blend proportions: sucrose = 0.227, wheat germ = 0.409, casein = 0.227, corn root powder = 0.136. Within each figure: A: Sucrose, B: wheat germ, C: casein, and D: corn root.

### 2-component lipid mixture experiment

Response surface models for weight and survival were generated by varying 2 lipid components: wheat germ oil and linseed oil (Table 5). Models indicated that the 2 lipid components had a minor contribution on improving larval weight, survival and molting.

The linear model for survival was significant (*p* = 0.049). The model indicated that linseed oil had a positive effect while wheat germ oil had a slightly negative effect on larval survival (Fig 5). The best model for weight gain was the overall mean. Neither oil had an effect on weight.

**Fig 5:** Predicted survival plots for WCR larvae reared on diets that vary in lipid content. Red dots are predicted values by the model at 7 days post infestation. Dotted lines indicate 95% confidence interval bands. Regression equation: Survival = 0.99*Linseed oil + 0.73*Wheat germ oil.

The model for molting was not generated because few larvae molted to second instar during this experiment. Within the range of proportions tested, the 2 oil components did not improve molting from first to second instar.

### Contamination

There was minor contamination (<1%) during all experiments and all time points evaluated. Consequently, there was no evidence for a relationship between contamination and diet ingredients.

### Model evaluation and diet improvement

The diet optimization for WCR larvae produced a formulation, referred to hereafter as WCRMO-1 (Table 6), that yielded better larval performance compared with the Pleau et al. diet (Table 7). WCRMO-1 was formulated in terms of maximizing an overall value of all three diet traits (survival, molt, and weight) simultaneously by optimizing the concentration of ingredients in the first WCR diet described by Pleau et al. [17]. At 7 days post infestation, there was a significant difference in survival rate between larvae reared on WCRMO-1 and on the Pleau et al. diet [17], but there were no significant differences in larval dry weight and molting rate. However, a significant improvement was seen in all three measures of larval performance at 11 days post infestation. At 11 days after infestation, the three measures (survival, molt, and weight) were significantly higher for larvae reared on WCRMO-1 compared with larvae reared on the Pleau et al. diet (Table 7). The level of improvement in larval dry weight gain was a two-fold increase and the survival and molting rate for larvae reared on WCRMO-1 were approximately 99%, compared to 93% and 90%, respectively when reared on the Pleau et al. diet.

**Table 6:** Diet formulation improvement for WCR development (109 g).

Ingredients	Pleau et al. (2002)	WCRMO-1
Sucrose	3.85 g	2.5 g
Wheat germ (raw, ground)	5.45 g	5.5 g
Casein	3.23 g	2.5 g
Cellulose	1.38 g	1.5 g
Corn root powder	0.63 g	1.5 g
Agar	1.45 g	1.5 g
Linseed oil, raw	40 μl	25 μl
Wheat germ oil	-	25 μl
Cholesterol	6 mg	6 mg
Wesson's salt mix	0.93 g	0.93 g
Vanderzant Vitamin mix	0.90 g	0.90 g
Methyl paraben	0.10 g	0.10 g
Sorbic acid	64 mg	64 mg
Potassium hydroxide (10%)	3.5 ml	3.5 ml
Streptomycin (12.8 mg/ml)	6.4 mg	6.4 mg
Chlortetracycline (10.0 mg/ml)	6.4 mg	6.4 mg
Distilled water	88 ml	88 ml
Green food coloring	64 μl	64 μl

**Table 7:** Larval dry weight, survival, and percent successful completion of molt for western corn rootworm larvae reared on WCRMO-1 and Pleau et al. [17] diets for 7 or 11 days.

	7 days			11 days		
	Weight	Survival	Molt	Weight	Survival	Molt
Diet	(μg)	(%)	(%)	(μg)	(%)	(%)
WCRMO-1	100 ± 3.1	99 ± 2.1 a	13 ± 5.9	425 ± 54.7 a	99 ± 1.8 a	99 ± 1.8 a
Pleau et al.	106 ± 16.1	91 ± 5.2 b	4 ± 3.4	196 ± 32.4 b	93 ± 4.7 b	90 ± 4.8 b

Means within columns followed by different letters are significantly different (α = 0.05, ANOVA). Mean ± SD.

## Discussion

The application of RSM based on a multivariate mixture design enabled us to concurrently evaluate several ingredients of an artificial diet for rearing WCR. By applying this method to a published formulation [17], we optimized 8 ingredients based on life history criteria (survival, molt, and weight). By applying good laboratory practices, as described above, we were able to decrease contamination and extend the assay period to 11 days and thereby measure events that had not occurred within shorter assay periods, e.g., molting and survival.

Results indicated that corn root powder, casein and wheat germ were key ingredients effecting larval performance, i.e., changing the concentration of these ingredients affected the life history parameters. In contrast, changing the proportion of other ingredients, including cellulose, sucrose, linseed oil, wheat germ oil and agar, had little or no negative effects on the response parameters.

We observed complex relationships between the response parameters and the proportionality of the key ingredients. Relatively small adjustments in the proportions of these nutrients resulted in a dramatic improvement in diet performance. As has been reported for other insect diets [38], we found an inverse relationship between weight, survival and molting as the proportions of corn root powder, casein, and wheat germ varied.

Corn root powder provided the most pronounced example of these complex relationships. Our results showed that corn root powder at high proportions improved molting and survival, but caused a decrease in weight when changed in combination with casein, wheat germ and sucrose. Pleau et al. (2002) reported a similar pattern in which corn root powder at high proportion did not yield larval weight gain with an OIAT design. An increase in proportion of corn root powder up to 0.6% (w/v) resulted in an increase in larval weight, but corn root powder at higher concentrations did not yield an increase in weight [17].

Our results indicated that casein also had a complex relationship with the life history parameters. Pleau et al. [17] documented that casein in the diet contributed significantly to WCR larval weight gain with an OIAT design. Cohen [26] suggested that an inclusion of the casein in diet mixtures may result in important interactions with other ingredients. Casein can reduce gel strength, possibly by reducing the capability of agar to bind water ([26], personal observation) or by binding calcium ions which may debilitate cross-linking in the gel matrix [39].

We also found a complex relationship between wheat germ and life history parameters. There was a direct correlation between the proportion of wheat germ and survival but at high proportions there was a negative effect on larval weight and molting. Pleau et al. [17] reported that an increase in wheat germ above 5.45% (w/v) had a negative effect on larval weight, but removal of wheat germ resulted in a significantly negative effect on WCR growth. Wheat germ is a key dietary component contributing to nutritional value, digestibility, bioavailability, and palatability, but at high concentrations can result in a deleterious effect on insect growth [26].

Contamination has been one of the limiting factors with diet when used to rear WCR and for toxicity-bioassays [14, 15]. Previously, microbial contamination (bacteria and fungi) forced diet bioassays to be terminated early and prevented more extensive observations. Typically, diet bioassays for rearing WCR ran for 6 days [17] while diet toxicity-bioassays ran for 4 to 7 days [18]. Those time points preceded 1^st^ to 2^nd^ instar molting. We were able to eliminate contamination through good laboratory practices which allowed for longer bioassays. By extending the bioassay to 11 days of feeding. we were able to detect differences among the formulations that were not detected at 7 days of feeding. For example, at 7 days WCRMO-1 and the Pleau et al. diet had similar larval performance. However, at 11 days larval performance on WCRMO-1 was better than the Pleau et al. diet (Table 7). At 11 days post infestation, larval dry weight, survival and molting rate of WCR larvae reared on WCRMO-1 were significantly higher than that of the Pleau et al. diet. Larval dry weight increased two-fold with WCRMO-1 as compared to the published diet. Survival and molting increased to approximately 99% with WCRMO-1.

WCR larval feeding typically ceases some hours before molting, and larval weight typically declines immediately following a molt ([40], personal observation). The improved performance in terms of weight gain of larvae reared on WCRMO-1 was particularly impressive in light of the greater proportion of those larvae that successfully completed the process of molting to the next instar compared with larvae reared on the Pleau et al. diet [17].

The goal of an artificial diet should always be to produce insects that develop similar to those reared on their natural food source [27]. WCR larvae molted at 7 days post infestation on maize [41]. However, only 12.5% WCR larvae molted to second instar at 7 days. when reared on WCRMO-1. While this is a major improvement over previous diets, and provides a diet suitable for toxicity bioassays (unpublished data, Hibbard/Coudron labs), these accomplishments also suggest additional formulation refinement may be possible and that a suitable substitution for corn root powder, which is not available from a commercial source, would be highly advantageous.
